The article "Empirical Analysis for Stock Price Prediction Using NARX Model with Exogenous Technical Indicators" was published in 2022. Journal: Comput Intell Neurosci.

# Empirical Analysis for Stock Price Prediction Using NARX Model with Exogenous Technical Indicators

**DOI:** 10.1155/2022/9208640

**Published:** 2022-03-25

**Authors:** Ali H. Dhafer, Fauzias Mat Nor, Gamal Alkawsi, Abdulaleem Z. Al-Othmani, Nuradli Ridzwan Shah, Huda M. Alshanbari, Khairil Faizal Bin Khairi, Yahia Baashar

**Affiliations:** ^1^Faculty of Economics and Muamalat, Universiti Sains Islam Malaysia (USIM), Bandar Baru Nilai, 71800 Nilai, Negeri Sembilan, Malaysia; ^2^Faculty of Computer Science and Information Systems, Thamar University, Thamar, Yemen; ^3^Cyber Technology Institute (CTI), De Montfort University, Gateway House, Leicester LE1 9BH, UK; ^4^Department of Mathematical Sciences, College of Science, Princess Nourah bint Abdulrahman University, P.O. Box 84428, Riyadh 11671, Saudi Arabia; ^5^Faculty of Computing and Informatics, Universiti Malaysia Sabah (UMS), Labuan, Malaysia

## Abstract

Stock price prediction is one of the major challenges for investors who participate in the stock markets. Therefore, different methods have been explored by practitioners and academicians to predict stock price movement. Artificial intelligence models are one of the methods that attracted many researchers in the field of financial prediction in the stock market. This study investigates the prediction of the daily stock prices for Commerce International Merchant Bankers (CIMB) using technical indicators in a NARX neural network model. The methodology employs comprehensive parameter trails for different combinations of input variables and different neural network designs. The study seeks to investigate the optimal artificial neural networks (ANN) parameters and settings that enhance the performance of the NARX model. Therefore, extensive parameter trails were studied for various combinations of input variables and NARX neural network configurations. The proposed model is further enhanced by preprocessing and optimising the NARX model's input and output parameers. The prediction performance is assessed based on the mean squared error (MSE), R-squared, and hit rate. The performance of the proposed model is compared with other models, and it is shown that the utilisation of technical indicators with the NARX neural network improves the accuracy of one-step-ahead prediction for CIMB stock in Malaysia. The performance of the proposed model is further improved by optimising the input data and neural network parameters. The improved prediction of stock prices could help investors increase their returns from investment in stock markets.

## 1. Introduction

The importance of the stock market to the international economy is undeniable [1]. Stock markets play a critical role in accelerating the growth of various sectors of the economy by facilitating the transfer of money from those with funds to those with the ability to invest it [2].

The article "Empirical Analysis for Stock Price Prediction Using NARX Model with Exogenous Technical Indicators" was published in 2022. Journal: Comput Intell Neurosci.

Wang et al. stated that different arguments had been made between participants in the market about the stock price predictability [3], with two arguments constituting the main ones. The first argument advocates that predictability is not possible because stock markets are efficient and future price movements are independent of past price action. The second argument argues that the market can be predicted or that its predictability can fluctuate between high and low levels.

Two hypotheses are closely related to the first argument regarding the unlikelihood of correct prediction, namely the Random Walk Hypothesis (RWH) and the Efficient Market Hypothesis (EMH). The RWH was introduced by [4], who stated who stated that future stock price values or directions could not be predicted based on past performance since stock price fluctuations are unrelated to one another. The EMH [5] implies that in an efficient market, all readily available information is incorporated, and stock prices respond to new information rapidly. Consequently, this rapid adjustment of stock prices in response to new information is frequently unanticipated, making the shift random [6]. Similarly, in [7], the study explains that the stock price follows a random walk behaviour because the market is efficient, and therefore, the movements of stock prices are unpredictable. Based on the multiple information levels (historical prices, public information, and private information) incorporated into the stock price, [5] categorised market efficiency into three types: weak-form EMH, semi-strong form EMH, and strong-form EMH. On the other hand, the Adaptive Market Hypothesis (AMH) introduced by [8] suggests that market efficiency is not fixed and can fluctuate between different efficiency levels. Market change is commonly driven by predictable investor behaviour, such as overconfidence, loss aversion, and overreaction. These investors' behaviours are consistent with human behavioural principles such as adaptation, competition, and natural selection [8, 9]. Therefore, AMH proposes that market efficiency and inefficiencies coexist in an intellectually consistent manner [10]. AMH can describe the predictability of major global stock indices where stock price predictability fluctuates with the time between periods of high predictability and other periods of low predictability, indicating that market efficiency is not an all-or-none situation [11].

Previous studies have attempted to predict the stock price or return movement with varying degrees of success (for example, [12–14]). Surveys conducted by [15] showed promising forecast results using conventional or digital computing models.

The article "Empirical Analysis for Stock Price Prediction Using NARX Model with Exogenous Technical Indicators" was published in 2022. Journal: Comput Intell Neurosci.

Accurate prediction of the stock market is still a big challenge because of the complexity and stochastic nature of the market data [16–21]. Specifically, the Malaysian stock market is a growing emerging market characterised by asymmetrical dynamic behaviour and weak market efficiency [22, 23]. Several studies were carried out to improve the prediction accuracy of different stock prices in Malaysia using various computational intelligence techniques [24, 25].

This paper's main objective is to analyse and compare the performance of the NARX neural network model to the performances of two other models [26, 27]. These models used the Feedforward Neural Network (FFNN) and Ensembled Feedforward Neural Network (ENN) models with macroeconomic variables in forecasting the CIMB stock market closing price. The CIMB stock is chosen as it was used in the [26, 27] models, and such selection was based on the fluctuation in the CIMB price data [26, 27].

This study explores the potential improvement in prediction performance by utilising technical variables in NARX models with optimised input data, preprocessing, and model parameter configuration. A comprehensive set of parameter trails for different combinations of input variables and different NARX neural network settings are investigated.

The remaining sections of the paper are organised as follows: Section 2 provides background on prediction techniques as well as an overview of notable studies on the subject. NARX's approach, experimental setup, and settings are all explained in Section 3.  Section 4 discusses and compares the experimental results, and finally, Section 5 draws the main conclusions of this study.

## 2. Literature Review

Forecasting the stock market is made by utilising a variety of prediction models. These forecasting models take technical and fundamental factors into account and as such, fundamental and technical analyses are two methods for forecasting a stock's future direction.

The fundamental analysis utilises economic and financial data about the company (e.g., revenue, workforce, infrastructure, and profitability) to determine the company's intrinsic value [28]. Fundamental analysis assumes that the market is logical, and the stock price depends on the company's real value and so, the price will eventually move towards the real (intrinsic) value.

On the other hand, forecasting stock prices can be accomplished by examining previous price and volume trends [29]. Thus, in technical analysis, characteristics such as peaks, bottoms, trends, and patterns all contribute to determining the stock's future value [28]. The main advantages of fundamental analysis are its structured evaluation and it offers superior long-term performance [30]. However, technical analysis might better predict the stock prices in the short-term [31–33], which is why traders frequently employ technical analysis [28]. Nevertheless, technical analysis is still criticised for its very subjective interpretation [34].

The article "Empirical Analysis for Stock Price Prediction Using NARX Model with Exogenous Technical Indicators" was published in 2022. Journal: Comput Intell Neurosci.

Researchers employed various conventional and digital computing prediction models. These models may incorporate different explanatory input variables from the fundamental and technical analysis [35]. The CAPM (Capital Asset Pricing Model) [36] is a well-known example of a conventional structural model [37]. CAPM describes the relationship between stock return including its risk and market return. The Arbitrage Pricing Theory (APT) expanded the relationship and described the relationship between a stock return and some macroeconomic variables [38, 39].

Other structural models can be classified as linear or nonlinear. Linear models include the linear-trend prediction model [40] and the exponential smoothing model, which assigns exponentially decreasing weights for time series prediction [41]. Additionally, the Autoregressive Integrated Moving Average (ARIMA) model gained momentum and is still widely regarded as a significant contribution to time series prediction. A key shortcoming of linear models is their inability to capture nonlinear trends in the data. Nonlinear models, such as GARCH (Generalized Autoregressive Conditional Heteroscedasticity), address this issue.

Some research suggests that nonlinear models might outperform linear models [42]. However, these studies are not conclusive and do not exclude the possibility that the opposite might occur [43].

Several studies have utilised the recent advancements in soft computing techniques and artificial intelligence to improve prediction model performance in forecasting the stock market [20, 24]. Soft computing methods for stock price prediction can capture and better handle the stock market's uncertain, noisy, and nonlinear patterns. Recently, these techniques have become more popular as they give a more accurate stock market prediction [44]. Artificial neural networks (ANNs) are soft computing models that mimic basic human brain processes in the central nervous system [44, 45]. The architecture of neural networks can be divided into different categories depending on the neuron's network layers and positions [46].

Various ANN training algorithms are available, each with its own benefits and drawbacks. Levenberg–Marquardt (LM), Bayesian Regularization (BR), and Scaled Conjugate Gradient (SCG) are three training algorithms that have been utilised successfully for stock market data prediction in prior studies [47–49].

The article "Empirical Analysis for Stock Price Prediction Using NARX Model with Exogenous Technical Indicators" was published in 2022. Journal: Comput Intell Neurosci.

The characteristics of the problem to be solved influence the choice of an ANN model. The feedforward neural network, for example, may not perform well if the input data pattern changes over time. A viable solution is to utilise a recurrent neural network (RNN), in which neurons have additional connections to the prior layer [50, 51].

This study employs a nonlinear autoregressive network with exogenous inputs (NARX), a type of recurrent neural network with high prediction capabilities for time series data. Given that the stock price prediction problem incorporates historical data as well as external variables, the NARX could be a compelling choice for modelling such a problem [49, 52–57].

A comparison of the prediction performance of the NARX model with other neural network models for the Indonesian stock index was carried out by [58] over a five-day forecasting period. The NARX model outperforms other neural network models' mean square error (MSE) performance. Similarly, in [53] research, predicting the NASDAQ closing price using a NARX prediction model outperforms other models such as VAR (vector autoregressive), ARIMA, and LSTM models.

In another recent study, Gandhmal and Kumar employed the NARX model to forecast the stock market using some technical indicators as exogenous variables. The NARX model outperformed a regression model, a Deep Belief Network (DBN) model, and a NeuroFuzzy model in terms of MSE and MAPE errors.

Moreover, Nikoli et al. (2019) suggest that the NARX model might successfully predict other financial time series data, such as the EUR/USD currency exchange rate. The prediction results can be enhanced further by integrating additional input variables and fine-tuning the NARX model's internal parameters [59].

## 3. Methodology

The main objective of this study is to compare and analyse the performance of an adaptive nonlinear autoregressive exogenous (NARX) neural network model that incorporates lagged pricing and technical indicators with two previously published models [26, 27]. The design of a neural network model for forecasting is a challenging endeavour due to the large number of parameters that may be altered to affect the performance of the ANN. Some of these parameters are associated with the selection and preprocessing of input data. Additional parameters related to neural network architecture include the number of hidden layers, the number of neurons, and the training algorithm. Furthermore, evaluation of the neural network requires selecting some performance measures.

The article "Empirical Analysis for Stock Price Prediction Using NARX Model with Exogenous Technical Indicators" was published in 2022. Journal: Comput Intell Neurosci.

This section discusses the experimental setup, including the model parameters used to perform the experiments. The first step is to collect data on CIMB stock and then compute the technical factors. After that, the data is filtered and normalised during the preprocessing stage. The data is then partitioned into input and test sets, which are then fed into the NARX neural network model.

Following that, the prediction model is constructed, and its parameters are adjusted, after which the model is put through a series of trials to determine its performance. Finally, all experiments' output results are saved for further evaluation and comparison. The overall methodology is depicted in Figure 1, and the subsequent sections describe each stage in further detail.

### 3.1. Data Collection and Preprocessing

The NARX model input data includes the CIMB stock adjusted closing prices and three-day lagged data, as well as six calculated technical variables: momentum, MACD, RSI, oscillator, WPCTR, and CHVOL. For technical factors (refer to Table 1), an arbitrary combination is used in the experiments because no prior knowledge exists regarding which combination will perform better.

CIMB stock data was obtained from the Yahoo Finance website for a ten-year period (2^nd^ Jan., 2008 to 29^th^ Dec., 2017). Two thousand three hundred thirty-three observations were included in the CIMB stock information dataset (trading days). Each observation included daily data on the lowest and highest prices, the opening and closing prices, and trading volume. Based on this, three subsets of the ten-year dataset were constructed (five years, three years, and one year).

After collecting the data, it was analysed to identify and eliminate any missing or erroneous values. Observations with missing, zero, or null closing prices correspond to days when no trading happens due to weekends, holidays, or other events, and these were all excluded from the datasets. Technical indicators are calculated during the preprocessing stage, and the data is subsequently normalised and smoothed, as described below.

#### 3.1.1. Calculating Technical Variables

Six technical indicators for the CIMB stock were calculated using the collected data. The following are the technical indicators that were chosen and their formulas:

*(1) Momentum (MOM)*. This indicator recognises price movement in terms of strength and speed by measuring the price (P) change rate. It is calculated by determining the difference between the current and past prices over an n-period.

(1) $$\begin{array}{c} {\text{MOM}}_{t}=P_{t}-P_{t-n}. \end{array}$$

In the calculation, the frequently adopted value of *n*=12[50] is used. In MATLAB, MOM is calculated using the built-in function tsmom.

*(2) Moving Average Convergence Divergence (MACD)*. Another momentum indicator for trending stock price data is MACD. It depicts the relationship between two stock price moving averages (the 26th and 12 day exponential moving averages) [60]. The macd MATLAB function is used to calculate MACD.

*(3) Relative Strength Index (RSI)*. The relative strength index (RSI) measures the magnitude and velocity of stock price changes [60]. RSI is computed in MATLAB using the rsindex function.

*(4) On-Balance-Volume (OBV)*. OBV measures stock momentum by relating volume and stock price changes [60]. The onbalvol function in MATLAB is used to calculate OBV.

*(5) Williams' Percent Range (Williams' %R) or (WPCTR)*. This technical indicator is used to determine whether or not a stock is oversold or overbought in the market [60]. The calculations in this study were based on a 14 day period. WPCTR % *R* is calculated in MATLAB using the willpctr function.

*(6) Chaikin Volatility (CHVOL)*. CHVOL is used to compare the spread between a stock's high and low prices by quantifying the volatility based on the changes of the moving average over a specific period. In this study, MATLAB's chaikvolat function was used to calculate CHVOL.

The article "Empirical Analysis for Stock Price Prediction Using NARX Model with Exogenous Technical Indicators" was published in 2022. Journal: Comput Intell Neurosci.

#### 3.1.2. Normalization and Smoothing

After calculating the technical indicators, the data is preprocessed using the smoothing and normalisation transformation techniques to improve the prediction outcomes [46]. The CIMB adjusted closing price data was smoothed using a five-day Exponential Moving Average (EMA) to minimise daily data's noisy and erratic effects. Then the input data that includes the smoothed CIMB stock's adjusted closing price and the calculated technical indicators are normalised to zero mean and unit variance [50].

### 3.2. Building the Prediction Model

This study employed a single-layered neural network structure of a nonlinear autoregressive exogenous (NARX) model. The NARX model uses a single hidden layer because single-layer models often give better prediction results and are more practical due to their ability to reduce computation time and reduce the risk of overfitting, which can degrade prediction performance [50, 61].

The following steps describe how the NARX model's parameters were set and optimised in MATLAB.

#### 3.2.1. Selecting Initial Model Parameters

The absence of a systematic method for determining the appropriate quantity of inputs that can affect the learning performance of neural networks is unfortunate [42]. Consequently, numerous parameters were investigated and tested in this study to optimise model performance, including the following:

*(1) Data size*. CIMB closed price data for (one, three, five, and ten) years.

*(2) Inputs*. The model's inputs are CIMB closing price data and exogenous variables (technical factors), which were combined in arbitrary combinations by adding one variable at a time. No variable switching was performed between exogenous variables, as this would significantly complicate the experiments. Additionally, the model was supplied with lagged data of the CIMB closing price and the exogenous variables. The number of lags varied; both the closing price and exogenous input lags ranged between 0 and 3.

*(3) Data split*. Two datasets were created from the input data. The first 90% of data was utilised as the neural network's input dataset, while the remaining 10% was unknown to the model and was used as a testing dataset and not for training. The 90% input dataset was then split into three segments, 70% training data, 15% testing data, and the remaining 15% was validation data (see Figure 2). The data split used in this arrangement was chosen based on the author's work [50].

The article "Empirical Analysis for Stock Price Prediction Using NARX Model with Exogenous Technical Indicators" was published in 2022. Journal: Comput Intell Neurosci.

#### 3.2.2. Determining the Best Number of Neurons

In the neural network design process, the number of input and output neurons is chosen based on the data used to solve the problem (i.e., the input features and outputs). There is no consensus on the optimal number of hidden neurons although some literature gives rules of thumb that can be utilised as a jumping-off point for experiments. The use of a fixed technique, in which the number of hidden neurons is changed while keeping all other parameters constant, can be used to identify the optimal number of neurons, resulting in the minimization of errors, the prevention of overtraining, and the avoidance of local minima. During the training phase, this study optimised by using a variety of different numbers of neurons. The range of neurons employed in the search for the optimal number of neurons was based on [50, 62], in which the maximum number of neurons is determined by the number of inputs and outputs as stated in equations (2) or (3).

(2) $$\begin{array}{c} \text{No.of neurons}=2\times \text{no.of inputs}+1, \end{array}$$

(3) $$\begin{array}{c} \text{no.of neurons}=\sqrt{n_{i}}\times \sqrt{n_{o}}, \end{array}$$

where *n*_*i*_  = number of inputs, *n*_*o*_  = number of outputs.

#### 3.2.3. Determining the Best Neural Network

Different parameter combinations were tested in order to identify the optimal neural network for the study model in terms of prediction accuracy as measured by mean square error (MSE). Three different training algorithms were used with both the training and testing sets, including the Levenberg–Marquardt algorithm (trainlm), Bayesian Regularization (trainbr), and Scaled Conjugate Gradient (trainscg).

The article "Empirical Analysis for Stock Price Prediction Using NARX Model with Exogenous Technical Indicators" was published in 2022. Journal: Comput Intell Neurosci.

The Leveneberg Marquardt algorithm (LM) is a more powerful optimization than the gradient descent [61, 62]. It outperforms both conjugate gradient and variable learning rate algorithms in neural networks of moderate size [63]. Bayesian Regularization is a training technique that updates the weight and bias values using Levenberg–Marquardt optimization. It minimises a combination of square errors and weights and determines the ideal combination for constructing a well-generalized network [64]. The scaled conjugate gradient algorithm (SCG) was introduced by [65] as a rapid training algorithm that removes the time spent online searches and combines the conjugate gradient and model-trust region approaches. These three training algorithms were identified to be dominant training algorithms in the stock market prediction field, with exceptional performance [48, 49, 66].

The random initialization of biases and weights is another issue to consider when designing neural networks, as two networks with identical designs and parameters might generate different results (Fang et al., 2014). This issue was addressed in this study by training many networks and picking the one with the lowest mean square error.

Moreover, to avoid overfitting, the neural network is first trained on a large part of the data sample and then tested on the remaining, smaller part to see if it can generalise what it learned during training when met with unknown data.  Figure 3 compares the model's performance on both in-sample and out-of-sample forecasts in terms of adjusted *R*^2^.

#### 3.2.4. Setting UP the Model

After setting the initial model parameters and selecting the optimal number of neurons and neural network, the final model is constructed and prepared for testing with various combinations of exogenous factors and input dataset durations.

### 3.3. Running and Evaluating the Model

#### 3.3.1. Running the Model

Three cascading loops were utilised to run the model and test all potential combinations efficiently. The first loop modifies the amount (duration) of data inputs (one year, three years, five years, and ten years). The second loop is responsible for selecting the training algorithms (trainlm, trainbr, and trainscg). Finally, the third loop selects various exogenous variable combinations (technical factors). In each iteration of these loops, the model is run on the training dataset then the test dataset.

#### 3.3.2. Performance Evaluation

The test data was used to evaluate the model's performance using three widely used performance metrics: mean square error (MSE), hit rate (HR), and R-squared coefficient of determination (*R*^2^) [27, 67] (Gan et al., 2019). These three metrics were computed for the training and testing datasets, respectively.

The article "Empirical Analysis for Stock Price Prediction Using NARX Model with Exogenous Technical Indicators" was published in 2022. Journal: Comput Intell Neurosci.

MSE is dependent on the data type and order of magnitude and is calculated as follows:

(4) $$\begin{array}{c} MSE=\frac{1}{N}\overset{N}{\underset{i=1}{\sum }}{\left({\bar{x}}_{i}-x_{i}\right)}^{2}, \end{array}$$

where *x*_*i*_ denotes the actual data for the *i*^*th*^ observation (out of *N* observations), and ${\bar{x}}_{i}$ denotes the model forecasted data.

Hit rate (HR) measures the prediction accuracy by calculating the percentage of correct movement of the predictions either up or down.

The *R*^2^ (R-squared coefficient of determination) is also used to indicate the prediction accuracy as it measures the percentage of the response variable variation explained by the model [68]. *R*^2^ is calculated using the following equation:

(5) $$\begin{array}{c} R^{2}=1-\frac{\sum_{i=1}^{n}{\left({\hat{y}}_{i}-y_{i}\right)}^{2}}{\sum_{i=1}^{n}\left(y_{i}-\bar{y}\right)}, \end{array}$$

where *n* denotes the total number of data points, $\hat{y}$ denotes the predicted value and $\bar{y}$ denotes the average value of actual output, and *y*_*i*_ denotes the actual output [69].

## 4. Results and Discussion

A total of 72 experiments were conducted to evaluate the developed ANN-NARX model's performance in predicting the CIMB stock closing price, with each experiment incorporating a different combination of data size (duration), exogenous variables (technical indicators), training functions (algorithms), and the optimal number of neurons. As stated in Table 1, the following six technical indicator combinations were employed in these experiments:

Tables 2–5 summarise the performance of the proposed NARX model in these experiments, utilising both training and testing datasets.

The model performance results reveal that the proposed model performs remarkably well in predicting the CIMB stock adjusted closing price movement. The model achieved a high hit rate percentage that reaches above 81% with a low average MSE of 0.000618044, which indicates that the average error of the proposed model is as low as $\sqrt{0.000618044}=0.02486$ Malaysian Ringgit. The proposed NARX model's accuracy (in terms of *R*^2^) ranged from 97.21% to 99.88%.

The proposed model performed best in terms of hit rate (HR) in experiment 22 (HR = 81.25%), where three years of data were used as input, technical factors (MOM, MACD, RSI, and OBV) were utilised as exogenous variables, and (trainlm) was used as the training function.

Figure 4 shows that the one-year duration performed lower than the other durations in terms of average MSE and average hit rate, which could be attributed to the model being trained on an inadequate amount of historical data to provide accurate predictions. The model's performance significantly improved as the amount of data used as input was raised to three years. However, there was no evidence of a significant improvement in the model's performance when the data set was increased to five and ten years.

The article "Empirical Analysis for Stock Price Prediction Using NARX Model with Exogenous Technical Indicators" was published in 2022. Journal: Comput Intell Neurosci.

As for the training algorithms illustrated in Figure 5, the Levenberg Marquardt algorithm (trainlm) and Bayesian Regularization (trainbr) both displayed slightly higher performance (in terms of average MSE) when compared to the Scaled Conjugate Gradient (trainscg) algorithm. On the other hand, the (trainlm) algorithm achieved the best overall averages in both MSE and Hit Ratio.

Regarding the number of neurons in the neural network, as indicated in Figure 6, the highly fluctuating results indicate that the number of neurons has no definitive effect on the model performance.

Additionally, Figure 7 shows that the combination of exogenous factors (MOM, MACD, and RSI) achieved the lowest MSE result. Increasing the number of technical factors in the prediction model had little effect on the *R*^2^ while degrading the average MSE and hit rate.

Furthermore, it was also noticed that adding more exogenous variables was only helpful when the data duration is longer than a year. However, when a longer duration was paired with more technical indicators, as illustrated by combining Figures 5 and 6, the performance was generally degraded in terms of the average MSE.

### 4.1. Model Performance Compared to Prior Studies

As shown in Table 6, the proposed NARX-model significantly increased forecast accuracy in terms of mean square error (MSE) when compared to the model proposed by [26, 27]. The proposed model's best and mean MSE values are lowered to (0.0003955) and (0.000618044), respectively, compared to (0.02198) for the best and (0.03149) for the mean MSE in [26, 27]. This improvement could be attributed to incorporating technical factors and preprocessing, which includes data smoothing using moving averages and optimization of the proposed model's parameters.

## 5. Conclusion and Future Work

In this study, the problem of stock market prediction is examined for a selected stock on the Malaysian stock exchange. The prediction of the CIMB stock closing price one step ahead was investigated using technical variables in a NARX neural network. The prediction performance was improved by including technical variables as exogenous inputs to the model, preprocessing the input data, and optimising the neural network's input variables and parameters. The model proposed in this study outperformed two other models previously published in the literature in terms of hit rate and MSE.

The article "Empirical Analysis for Stock Price Prediction Using NARX Model with Exogenous Technical Indicators" was published in 2022. Journal: Comput Intell Neurosci.

The results suggest that including technical indicators into the NARX neural network model has a high potential for improving prediction performance and is demonstrated by examining performance indicators such as MSE, Hit rate, and *R*^2^.

In this study, only three training algorithms (trainlm, trainbr, and trainscg) were examined. To further improve prediction performance, it may be useful to investigate other widely used training algorithms such as, gradient descent and gradient descent with momentum in future studies.

Additionally, this study only considered the use of technical indicators as exogenous variables in the NARX model arbitrarily for only one stock in the Malaysian stock market. In future works, it might be beneficial to optimise the selection of the exogenous variables by using advanced features selection methods such as, deep mining and exploring the use of integrating fundamental factors to improve the prediction for different stocks in the market.

## Figures and Tables

**Figure 1:** Methodology and research phases.

**Figure 2:** Splitting of input data.

**Figure 3:** Adjusted *R*^2^ for in-sample and out-of-sample forecasts.

**Figure 4:** Performance based on dataset length (duration).

**Figure 5:** Performance based on training function.

**Figure 6:** Performance based on number of neurons.

**Figure 7:** Performance based on the technical indicators.

**Table 1:** Technical indicators combinations.

Set	Exogenous variables
Set A	(MOM)
Set B	(MOM, MACD)
Set C	(MOM, MACD, RSI)
Set D	(MOM, MACD, RSI, OBV)
Set E	(MOM, MACD, RSI, OBV, WPCTR)
Set F	(MOM, MACD, RSI, OBV, WPCTR, CHVOL)

**Table 2:** Performance results of the proposed NARX model (1 year dataset).

Algo.	Technical indicator set	Best no. Of neuron	In-sample forecasting (training data)			Out-of-sample forecasting (testing data)		
			MSE	Hit rate (%)	Adj *R*^2^ (%)	MSE	Hit rate (%)	Adj *R*^2^ (%)
Trainlm	A	2	0.00041966	79.79	99.85	0.00098469	76.19	97.58
	B	3	0.00044278	80.85	99.84	0.00087177	76.19	97.84
	C	3	0.00043388	79.79	99.85	0.00095494	66.67	97.72
	D	5	0.00036067	77.66	99.87	0.0010599	80.95	97.50
	E	4	0.00041745	77.66	99.86	0.00095836	76.19	97.80
	F	4	0.00037631	79.79	99.87	0.0010421	71.43	97.48

Trainbr	A	2	0.00039668	80.32	99.86	0.00089625	71.43	97.84
	B	9	0.00039637	81.38	99.86	0.00097039	71.43	97.67
	C	11	0.00038865	79.26	99.86	0.00097508	76.19	97.68
	D	13	0.0003833	78.72	99.86	0.00098283	71.43	97.61
	E	20	0.00040986	80.32	99.86	0.00093343	66.67	97.70
	F	16	0.00038355	80.32	99.87	0.0008733	66.67	97.84

Trainscg	A	4	0.00043191	80.32	99.85	0.00093434	71.43	97.70
	B	13	0.000493	76.06	99.83	0.0011909	71.43	97.21
	C	7	0.00044605	79.79	99.84	0.00081055	80.95	98.06
	D	5	0.00045183	80.85	99.84	0.0010654	80.95	97.47
	E	6	0.0004218	79.26	99.85	0.00094762	71.43	97.66
	F	4	0.00053291	74.47	99.81	0.00101	61.90	97.49

The article "Empirical Analysis for Stock Price Prediction Using NARX Model with Exogenous Technical Indicators" was published in 2022. Journal: Comput Intell Neurosci.

**Table 3:** Performance results of the proposed NARX model (3 years dataset).

Algo.	Tech.Ind.s	Best no. of neuron	In-sample forecasting (training data)			Out-of-sample forecasting (testing data)		
			MSE	Hit rate (%)	Adj *R*^2^ (%)	MSE	Hit rate (%)	Adj *R*^2^ (%)
Trainlm	A	2	0.00069605	73.62	99.89	0.00045192	75.00	97.74
	B	3	0.00063624	74.14	99.90	0.00044785	79.69	97.79
	C	13	0.00059232	73.28	99.91	0.00039547	79.69	98.08
	D	3	0.00065832	73.79	99.90	0.0004582	81.25	97.75
	E	4	0.00068018	73.62	99.90	0.00053326	78.13	97.33
	F	4	0.00065302	75.00	99.90	0.00048444	76.56	97.68

Trainbr	A	2	0.00061839	75.00	99.90	0.00044037	76.56	97.81
	B	11	0.00061491	75.17	99.90	0.00043917	76.56	97.82
	C	3	0.00060378	73.62	99.91	0.00044144	78.13	97.82
	D	15	0.00060703	74.14	99.91	0.00047402	76.56	97.66
	E	24	0.00059912	74.66	99.91	0.00046232	78.13	97.74
	F	16	0.00060037	73.79	99.91	0.00047527	78.13	97.65

Trainscg	A	2	0.00077806	71.72	99.88	0.00053703	75.00	97.33
	B	9	0.00065653	75.17	99.90	0.0004329	78.13	97.86
	C	9	0.00067279	74.48	99.90	0.00041738	78.13	97.92
	D	3	0.00067804	75.34	99.89	0.00052069	78.13	97.42
	E	6	0.00070628	71.55	99.89	0.00053084	70.31	97.35
	F	4	0.00068388	74.31	99.89	0.00050886	76.56	97.46

**Table 4:** Performance results of the proposed NARX model (5 years dataset).

Algo.	Tech. Ind.s	Best no. of neuron	In-sample forecasting (training data)			Out-of-sample forecasting (testing data)		
			MSE	Hit rate (%)	Adj *R*^2^ (%)	MSE	Hit rate (%)	Adj *R*^2^ (%)
Trainlm	A	4	0.00075225	74.43	99.93	0.0005291	75.93	98.93
	B	3	0.0007426	76.29	99.93	0.00048333	75.93	99.02
	C	3	0.00074319	75.26	99.93	0.00051512	74.07	98.97
	D	3	0.0007068	76.08	99.93	0.00057083	70.37	98.86
	E	4	0.00072597	75.46	99.93	0.00051831	71.30	98.96
	F	4	0.00071512	76.80	99.93	0.00056231	75.00	98.87
Trainbr	A	4	0.00070654	75.67	99.93	0.00045129	75.93	99.09
	B	3	0.00069784	76.08	99.93	0.00050233	78.70	98.99
	C	3	0.00068728	76.70	99.94	0.0005184	72.22	98.96
	D	3	0.00067918	75.77	99.94	0.00055092	71.30	98.88
	E	4	0.00061967	77.11	99.94	0.0007924	65.74	98.40
	F	30	0.00069623	75.15	99.93	0.00061321	71.30	98.76

Trainscg	A	8	0.00085249	71.75	99.92	0.00050295	74.07	98.98
	B	5	0.00074878	75.36	99.93	0.00050889	75.00	98.96
	C	5	0.00076245	76.29	99.93	0.00048381	73.15	99.02
	D	5	0.0007681	75.05	99.93	0.00054994	71.30	98.88
	E	4	0.0007747	73.81	99.93	0.00054574	75.00	98.88
	F	4	0.00082532	74.02	99.92	0.00058778	75.00	98.80

The article "Empirical Analysis for Stock Price Prediction Using NARX Model with Exogenous Technical Indicators" was published in 2022. Journal: Comput Intell Neurosci.

**Table 5:** Performance results of the proposed NARX model (10 years dataset).

Algo.	Tech.Ind.s	Best no. Of neuron	In-sample forecasting (training data)			Out-of-sample forecasting (testing data)		
			MSE	Hit rate (%)	Adj *R*^2^ (%)	MSE	Hit rate (%)	Adj *R*^2^ (%)
Trainlm	A	8	0.00062017	73.28	99.97	0.00045668	79.57	99.88
	B	5	0.00060706	73.90	99.97	0.00045396	79.57	99.88
	C	3	0.00059915	74.29	99.97	0.00045704	80.00	99.88
	D	5	0.00059822	74.29	99.97	0.00047444	77.39	99.88
	E	4	0.00063656	73.95	99.97	0.00048519	77.39	99.87
	F	6	0.0005966	73.37	99.97	0.00053886	78.26	99.86

Trainbr	A	2	0.00060374	74.05	99.97	0.00044822	80.43	99.88
	B	3	0.00059598	74.58	99.97	0.00045795	79.57	99.88
	C	3	0.00059492	74.05	99.97	0.0004652	78.26	99.88
	D	3	0.00059241	74.38	99.97	0.00047232	79.13	99.88
	E	4	0.00057363	74.34	99.97	0.00052785	76.96	99.86
	F	4	0.00057536	73.81	99.97	0.00053742	77.39	99.86

Trainscg	A	8	0.00069642	72.50	99.96	0.00048991	80.87	99.87
	B	13	0.0006516	73.90	99.97	0.00048468	77.83	99.87
	C	11	0.00070192	71.35	99.96	0.00051978	76.96	99.86
	D	5	0.00067275	72.74	99.97	0.00051608	78.70	99.87
	E	16	0.00063183	74.10	99.97	0.00048529	76.09	99.87
	F	8	0.0006567	74.24	99.97	0.00052833	77.83	99.86

**Table 6:** Comparison between the proposed model and two previously published models in literature.

	External constraints of neural cognition for CIMB stock closing price prediction [26]	Homogeneous ensemble feedforward neural network in CIMB stock price forecasting [27]	Current study
**Year**	2017	2019	2022
**Aim**	FFNN was used to forecast the CIMB stock closing price. The CIMB stock was selected due to its price fluctuation	Comparison between the performances of FFNN and a homogenous ensemble FFNN in forecasting CIMB stock market closing price	Comparison between the performance of NARX neural network to previous models
**Input data**	CIMB stock information (opening price, closing price, highest price, lowest price and volume trade), in addition to the exogenous variables	CIMB stock information (opening price, closing price, highest price, lowest price and volume trade), in addition to the exogenous variables	CIMB stock information (opening price, closing price, highest price, lowest price and volume trade), in addition to the exogenous variables
**Exogenous variables**	KLCI index, interest rate and currency exchange rates (USD, EUR, and SGD)	KLCI index, interest rate and currency exchange rates (USD, EUR, and SGD)	Technical indicators: Six combinations of technical indicators are used in these experiments: Set *A*= (MOM), set *B* = (MOM, MACD), set *C* = (MOM, MACD, RSI), set *D* = (MOM, MACD, RSI, OBV), set *E* = (MOM, MACD, RSI, OBV, WPCTR), and set *F* = (MOM, MACD, RSI, OBV, WPCTR, CHVOL).
**Period**	January 2000 and Jun 2015	January 2000 to June 2015	A 10 year (02-Jan-2008 to 29-dec-2017
**No. Of history day**	5	5	3 optimized to select the one with the lowest MSE
**Missing value**	The missing value is then derived by averaging the previous and next day's values.	If there is a missing value, this missing value is derived by averaging the previous and next day's values.	Not replaced, observation with missing value is deleted
**Normalization**	Yes	Yes	Yes
**Smoothing**	No	No	Five days exponential moving average (EMA) is used for the closing price.
**Training and testing**	The training (70%), validation (15%) and testing sets (15%)	The training (70%), validation (15%) and testing sets (15%)	Out of sample forecast on a 10% of the data The 90% input dataset is then split into three segments, 70% training data, 15% testing data (in-sample forecasting), and the remaining %15 is validation data.
**ANN architecture**	A single hidden layer FFNN model	A single hidden layer A homogenous ensemble FFNN model	A single hidden layer Recurrent networks (NARX model)
**No of hidden neurons**	(Input neurons + output neurons)/3	Selected based on a rule of thumb which is the number of input neuron plus number of output neuron divided by two(input neurons + output neurons)/2	Optimized. During the network's training phase, an optimization process employed a range of different neuron numbers.
**Training algorithm**	Levenberg–Marquardt algorithm	Levenberg–Marquardt algorithm	Levenberg marquardt algorithm (trainlm), bayesian regularization (trainbr), and scaled conjugate gradient (trainscg)
**Evaluation function**	MSE	MSE	MSE
**Lowest MSE FFNN**	Best MSE result = 0.03724 Mean MSE result = 0.03743	MSE FFNN model = 0.0201. MSE ENN model = 0.0193 Results showed that homogenous ensemble ANN performed better than a single ANN in predicting the stock market price.	The best and mean MSE results for the proposed model are reduced to 0.0003955 and 0.000618044, respectively
**Prediction accuracy hit rate**	N/A	FFNN = 58.1 ENN = 59.87	Best hit rate = 81.25%

The article "Empirical Analysis for Stock Price Prediction Using NARX Model with Exogenous Technical Indicators" was published in 2022. Journal: Comput Intell Neurosci.

## Data Availability

The data used to support the findings of this study are available from the corresponding author upon request.
